# Study of relationship between obesity and executive functions among high school students in Bushehr, Iran

**DOI:** 10.1186/s40200-015-0211-9

**Published:** 2015-10-15

**Authors:** Soqra Ebrahimi Qavam, Abbas Anisan, Marjan Fathi, Ata Pourabbasi

**Affiliations:** Faculty of psychology and education, Allameh Tabatabaee University, Tehran, Iran; Allameh Tabatabaee University, Tehran, Iran; Islamic Azad University, Kish Branch, Iran; Diabetes Research Center, Endocrinology and Metabolism Clinical Sciences Institute, Tehran University of Medical Sciences, 5th Floor, Sharitai Hospital, North Kargar Ave, Tehran, Iran

**Keywords:** Aobesity, Adolescents, Executive functions, Cognition

## Abstract

**Background:**

Obesity is one of the most challenging problems of public health in the present century and can have some serious impacts on cognitive abilities in children and adolescents. This study has tried to investigate the relationship between obesity and executive functioning, particularly in planning- organizing and problem solving among a group of adolescents.

**Methods:**

Some 120 male high school students in the 15 to 18 year age range were included. BMI and executive functions were measured with validetes tools and tests in cases.

**Results:**

There is a significant difference between the executive functions such as planning-organizing and problem solving in obese, overweight and normal students.

**Conclusions:**

According to our results it seems the obese adolescents have poorer executive functions than normal weight peers. This is important for families and school staff to design and follow some therapeutic plans for weight reduction in adolescents in order to help them improve their skills in some functions such as planning-organizing and problem solving.

## Introduction

Obesity as a widespread and prevalent disorder is causally associated with critical illnesses [1] and is one of the most challenging problems of public health in the present century. In addition, It is the most common nutrition - health problem in developed and developing countries which has great impact on many aspects of individuals and communities [2].

In general, the involvement of the health sector in the increasing incidence of complications remains relatively large yet, [3] including diabetes, coronary heart disease, hypertension, cerebrovascular diseases etc. [4]

According to Farzadfar et al. study on the epidemiology of obesity in 199 countries in 2008, there are 1.46 billion overweight and 502 million obese people in the world. [5] In Iran, approximately 19.4 % of adults are obese and 51.4 % are overweight.

Obesity is also linked to adverse neurodevelopmental outcomes such as degeneration of the frontal cortex and white matter brain damage [6]. In addition, recent studies have pointed to the link of obesity with poor cognitive functions [7]. Several studies have also reported degrees of cognitive vulnerability in obese subjects, including impairments in reaction time, alertness and attention, as well as immediate word recall, delayed recall, selective attention, processing speed and executive functioning, implicit memory, semantic memory and spatial abilities [8].

Executive functioning refers to a set of cognitive processes addressing the management of targeted behavior [9]. This ability is associated with the frontal lobe of the brain and the development of the prefrontal brain [10].

There are some controversies on whether the components of the executive functioning are affected by overweight and obesity in adolescents. This study has tried to investigate the relationship between obesity and executive functioning, particularly in planning- organizing and problem solving among a group of adolescents in Iran.

## Materials and methods

### Human subjects approval statement

This project was approved by the Ethical Board Committee of the Endocrinology and Metabolism Research Institute in accordance with Helsinki declaration and the guidelines of the Iranian Ministry of Health and Medical Education. All the students agreed to participate in the study.

### Participants

This observational study was carried out on 120 male high school students in the range of 15 to 18 year age including three groups of obese, overweight and normal students in Bushehr province of Iran in 2014.

### Measurement tools

#### Body mass index

The weight was measured at the minimum coverage and without shoes using a digital scale with a precision of 100 g. The height was measured via a stadiometer. The body mass index (BMI), the most commonly accepted index, was calculated to estimate obesity [11]. Based on the charts of the Reference Center for Disease Control, those having a BMI equal to or greater than the 95^th^ percentile for age and gender were considered as obese, and a BMI between 85 and 95 percentile for age and sex were taken as overweight [12].

#### Andre Rey test

Planning and organizing functions were measured by Andre Rey Test, which is standardized by Mir Hashemi in Iran [13]. The Test consisted of two cards, A and B, which were selected separately and in accordance with the situation. Card A included 18 cognitive components used for people aged four and older. The Effective performance of the card is for Seven year old children and older and more practical for teens and adults. [14].

#### Tower of London Test

It is the most famous test for the calculation of planning and problem solving. A computerized variant of this test was developed by Morris in which the vertebral ring with three-dimensional structure has been administered [15]. Two-tier arrangement is shown to participants on a screen touch computer. In each trial, top row remains constant and shows the arrangement of the target. The bottom row contains a loop that participants should rearrange it, so that it should match with the upper-tier arrangement. Target for the loop is variable, but the starting point is fixed. Minimum gestures through which the participants can solve the problem are 2, 3, 4, 5 movements [16]. Variables include total score, total run time, copy time and the number of errors [15]. The Correlation between the results of the test and Porteus Mazes has been reported as *r* =0.41 [17]. The validity of test (0.97) is accepted [18].

## Results

Students were matched according to their age, education and gender for the comparison of the executive functioning.

Descriptive parameters including frequency and percentage of subjects in each grade and age group are presented in Table 1. The mean and standard deviation (SD) in different groups of participants, Andrea Ray, Tower of London Tests are shown in Table 2.

**Table 1:** Demographic characteristics of samples of different groups

Demographic characteristics	Groups	Obese		Overweight		Normal	
		Number	Percent	Number	Percent	Number	Percent
School Grade	Junior high school	13	32.5	12	30	12	30
	second-grade high school	13	32.5	15	37.5	14	35
	third-grade high school	14	35	13	32.5	14	35
Age	15 years	14	35	13	32.5	12	30
	16 years old	13	32.5	13	32.5	14	35
	17 years	11	27.5	14	35	12	30
	18 years	2	5	0	0	2	5

**Table 2:** Descriptive characteristics of variables in obese, overweight and normal group

Groups	Obese			Overweight			Normal		
Variables	Numbers	M^a^	SD^b^	Numbers	M	SD	Numbers	M	SD
Planning- organizing first stage	40	35.15	1.05	40	35.85	1.08	40	35.77	1.26
Planning- organizing second stage	40	21.47	4.85	40	25.13	4.73	40	29.36	4.23
Tower of London total score	40	24.98	3.15	40	27.33	3.11	40	30.78	3.87
Tower of London runtime	40	440.90	176.57	40	387.25	165.57	40	275.07	149.57
Tower of London copy time	40	305.87	135.57	40	276.35	115.56	40	194.32	133.56
Tower of London errors	40	24.27	5.60	40	20.50	4.60	40	11.82	4.30

^a^mean

^b^standard deviation

Assumed to be normal, the distribution was examined by using the Kolmogorov-Smirnov one-sample test, and statistical significance of each variable was attained. Each variable was greater than 0.05 and the data on all variables were normal. (Table 3)

**Table 3:** Kolmogorov-Smirnov one-sample test

Statistics	Z	*P*	Significance level
Variables			
Planning-organizing first stage	0.83	0.51	0.05
Planning-organizing the second stage	1.22	0.09	0.05
Tower of London total score	1.24	0/09	0/05
Tower of London runtime	1.07	0.19	0.05
Tower of London copies	1.21	0.11	0.05
Tower of London errors	1.25	0.09	0.05

The homogeneity of variances was examined using Levine test. The significance level of the F-statistic in Levine test for London Bridge was greater than 0.05, so there was no significant difference between the group variance in the dependent variable which contributed to meeting the assumption of homogeneity of variances. The test statistics for Andre Ray is also greater than 0.05, Thus the analysis of homogeneity of variance test was performed in both groups and the results confirmed the assumptions. (Table 4)

**Table 4:** Levine F test for homogeneity of variance in three research groups

Variables	Tower of London errors	Tower of London copies	Tower of London run-time	Tower of London Total score	Planning, organizing the second round	Planning, organizing the first stage
Index						
df1^a^	2	2	2	2	2	2
df2	117	117	117	117	117	117
F	0.77	2/.1	0.35	0/18	0.02	0.05
sig	0.46	0.06	0.70	0.83	0.94	0.91

^a^Dgree of Freedom

After ensuring that all analyzed data were eligible using the analysis of variance, the test was performed. The multivariate analysis of variance was applied in order to compare the three groups in Planning Organization (Andre Rey test) and the solution (the Tower of London test). The results are reported In Tables 5 and 6.

**Table 5:** MANOVA and ANOVA test text

Statistical Indicators	Change sources	Ss^a^	df	F	Significance level	Effect size	Power of test
Variables							
Planning, organizing first phase	group	11.81	2	10.60	0.001	0.15	0.98
Planning, organizing the second phase	group	1246.36	2	38.65	0.001	0.39	0.99

^a^sum of squares

**Table 6:** MANOVA and ANOVA test

Statistical Indicators	Change resource	Ss^a^	df	F	Significance level	Effect size	Power of test
Variabes							
The Tower of London Total	Group	680.86	2	41.54	0.001	0.41	0.99
the Tower of London Runtime	Group	572793.12	2	18.52	0.001	0.24	0.99
the Tower of London Copy time	Group	267243.05	2	13.95	0.001	0.19	0.99
Tower of London Number of errors	Group	3260.12	2	55.25	0.001	0.48	0.99

^a^sum of squares

The obese, overweight and normal groups were compared using an Andre Ray test. The results of this analysis (Lambda = 0.48, Vickles, 0.05 > *P*, F (226, 10) -10/05), revealed the role of weight as an effective factor. These findings raised the issue that at least one component among three groups is different. The effect of weight for planning-organizing at the first and second stages is 0.15 and 0.13, which means that 15 % and 13 % of the variance of individual differences is related to weight. In addition, the statistical analysis suggested that the probability of correctly rejecting the null hypothesis of the test is at least 98%.

Table 6 shows the comparison of obese, overweight and normal subjects using the Tower of London. Considering the results of our analyses (Vickles Lambda = 0.43, *p* < 05/0, 98/14 = F (8 and 228) a significant effect of weight is appeared. These results indicated that at least one component of the problem solving (total score, runtime, copy and error) has some differences among normal, overweight and obese subjects. Afterwards, the significance level for each four problem solving subscales was obtained which was lower in comparison with which was obtained from the modified Bonferrony correction as 0. 15 (significance level split 0.05 of the 4 components of the problem solving).

In addition, the statistical analysis in this study suggested that the probability of the correctly rejection of the null hypothesis is at least 99 %. In order to accurately assess the difference between the three groups, the outcomes of the Tukey test showed that there is a significant difference in the total score of error and the numbers of subscales between the three groups.

## Discussion

In this study, we investigated the components of executive functioning, including planning-organizing and problem solving in obese, overweight and normal students. The results showed that there is a significant difference between the executive functions such as planning-organizing and problem solving in obese, overweight and normal students. These results are consistent with the findings of previous studies [7, 8, 19–27].

Fergenbaum et al. examined whether obesity is a predictor of decreased executive functioning and found out that poor performance of executive functions in obese people are five times more likely than healthy ones.[21] Also Fitzpatrick et al. in their study showed that obese individuals were weaker in decision-making, planning and problem solving compared to their normal weight peers [22]. However, MacGregor et al. showed in their study that there is no significant relationship between the obesity and cognitive functions after controlling for the relevant variables [28].

There are numerous definitions for executive functioning which include elements such as planning and purposeful, organized behavior over time, response inhibition, attention, working memory, self regulation processes, self-controlling and self monitoring [29]. These skills develop from childhood to adolescence and even to adulthood [30].

The above results can be explained by the relationship between obesity and adverse neurodevelopmental outcomes such as degeneration of the frontal cortex and white matter [6]. In fact, the underlying causes of obesity can be associated with the limbic neural circuitry destruction of orbital frontal cortex [31]. Since the ability of executive functioning is a part of the superior prefrontal cortex activity, it’s generally believed that the impairment or dysfunction of the prefrontal areas and some areas of the cerebral cortex are significantly associated with the student’s ability to perform executive functions [32]. Accordingly, it appears that the orbital frontal cortex and limbic circuit are associated with the prevention or reduction of the executive functions [33].

There are some possible biological mechanisms for the relationship between obesity and structural changes of the brain and its relevance with poor executive function. Obesity is highly correlated with the many changes that potentially can have a negative impact on cognitive functions like vascular changes such as thickening and hardening of the brain arteries, impaired insulin regulation, inflammation, cardiovascular disorders etc. [23].

Although the increased body mass index is along with decreased cognitive and executive functions, especially in the field of memory and executive functioning, problem solving and planning [7], but individuals with poor and impaired executive functioning are more likely to be overweight or obese. This may be due to the fact that many aspects of executive functioning such as impulse control, self and goal-oriented behavior is directly related to the ability to maintain energy balance [23].

The authors encountered some limitations in this study. The bureaucratic processes in the school setting hindered the cooperation of its administrators with researchers. On the other hand, considering that the evaluation of executive functions is still a new field in Iran and therefore few Persian literature are available. This study contains only two domains of executive functioning, including planning- organizing and problem solving in the Forum. We highly suggest that future researches also examine other executive functions among obese individual.

## Conclusion

According to our results, it can be concluded that the obese adolescents have poorer executive functions than normal weight peers. This is important for families and school staff to design and follow some therapeutic programs and interventions for weight reduction in adolescents in order to improve the executive functioning in them with the emphasis on the education of thinking and problem solving skills.
